# A Novel Memetic Algorithm Based on Multiparent Evolution and Adaptive Local Search for Large-Scale Global Optimization

**DOI:** 10.1155/2022/3558385

**Published:** 2022-03-24

**Authors:** Wenfen Zhang, Yulin Lan

**Affiliations:** ^1^School of Computer and Artificial Intelligence, Xiangnan University, Chenzhou, China; ^2^Hunan Engineering Research Center of Advanced Embedded Computing and Intelligent Medical Systems, Chenzhou, China

## Abstract

In many fields, including management, computer, and communication, Large-Scale Global Optimization (LSGO) plays a critical role. It has been applied to various applications and domains. At the same time, it is one of the most challenging optimization problems. This paper proposes a novel memetic algorithm (called MPCE & SSALS) based on multiparent evolution and adaptive local search to address the LSGO problems. In MPCE & SSALS, a multiparent crossover operation is used for global exploration, while a step-size adaptive local search is utilized for local exploitation. A new offspring is generated by recombining four parents. In the early stage of the algorithm execution, global search and local search are performed alternately, and the population size gradually decreases to 1. In the later stage, only local searches are performed for the last individual. Experiments were conducted on 15 benchmark functions of the CEC′2013 benchmark suite for LSGO. The results were compared with four state-of-the-art algorithms, demonstrating that the proposed MPCE & SSALS algorithm is more effective.

## 1. Introduction

Optimization problems widely exist in many fields such as engineering design, economic management, production scheduling [1–4], wireless communication, and computer science. Some of these problems have many decision variables that create Large-Scale Global Optimization (LSGO) problems. Without loss of generality, a large-scale global optimization can be formulated as a minimization problem as given in

(1) $$\begin{array}{c} \underset{x\in \text{Domain}}{\min}f\left(x\right),\text{Domain}\subseteq R^{D}, \end{array}$$

where *D* ≥ 1000 is the dimension size.

Large-scale global optimization is one of the most challenging optimization problems where the search space grows exponentially with increasing the problem dimensionality. Such a massive increase in problem dimensions usually changes the search properties. Consequently, the small-scale unimodal function may change to a multimodal function when the number of dimensions increases [5]. Therefore, researchers have proposed many improved algorithms based on the existing classic algorithms. For example, in [6,7], the Particle Swarm Optimization (PSO) algorithm was improved using subswarms to maintain diversity. Also, in [8], an improved PSO algorithm containing two types of learning strategies was provided. Multiple Offspring Sampling (MOS) [9] is a hybrid algorithm that combines a Genetic Algorithm (GA) and two local searches. MLSHADE-SPA [5] also is a hybrid algorithm that is based on three Differential Evolution (DE) strategies and a modified Multiple Trajectory Search (MTS) [10] algorithm. IMLSHADE-SPA [11] is an improved MLSHADE-SPA with a novel local search method. However, SHADE-ILS [12] is an enhanced version of the SHADE algorithm. It combines two different local search methods and uses a restart mechanism. Algorithms in [13–16] are modified algorithms based on Cooperative Coevolution (CC) and Differential Evolution. CBCC-RDG3 [17] is also a modified version of the CC algorithm that modifies the recursive differential grouping method to reduce the overlapping problems. TPHA [18] and DECC-RAG1.1 [19] are two-phase hybrid algorithms that use the CC framework.

To encourage the research on LSGO, IEEE Congress on Evolutionary Computation (IEEE CEC) organizes LSGO algorithm competitions yearly or biennial. Since 2013, it has been performed on the CEC′2013 LSGO benchmark suite [20]. MOS was the winner in the years 2013–2018. Moreover, MOS and the other 11 excellent algorithms that did not join the competitions were compared in [21]. Again, the MOS algorithm overperformed all the other algorithms. However, SHADE-ILS and MLSHADE-SPA were announced in the 2018 competition that they are performing better than MOS. Although CC-RDG3 [17] was announced as the winner of the 2019 competitions, it was not up to the level of the previous winner, SHADE-ILS. It seems that LSGO is still a quite hard nut to crack [21].

The algorithms for LSGO problems can be roughly classified into three categories: standard evolutionary algorithms, CC-based evolutionary algorithms, and memetic algorithms [22]. The memetic algorithm (MA) [23] is a combination of global search and local search. Due to the exploration ability of global search and the exploitation ability of local search, MA performs well in LSGO problems. As mentioned above, the CEC competition award algorithms (e.g., SHADE-ILS and MLSHADE-SPA) and improved algorithm IMLSHADE-SPA based on MLSHADE-SPA are all MAs. In MLSHADE-SPA, IMLSHADE-SPA, and SHADE-ILS, global search and local search have the same position, and the two search methods generate the same number of candidate solutions. However, since the dimension exceeds 1000 for LSGO problems, it is necessary to discuss the case that the numbers of local search and global search are different. Furthermore, at each iteration of the algorithms, the local search is only used to improve the current best solution, and other members cannot be improved, which may miss potential excellent individuals. Besides, the three algorithms all used Differential Evolution and adopted a variety of improvement strategies, which makes the algorithm more complicated. In this case, it is necessary to examine new algorithms and new ideas. This paper proposes a novel memetic algorithm (called MPCE & SSALS) based on multiparent evolution and local search. A multiparent crossover operator is used for global exploration. Furthermore, a step-size adaptive local search algorithm, which is improved from the MTS algorithm, is proposed for local exploitation. The proposed algorithm is inspired by the Simplified Group Search Optimizer (SGSO) [24] algorithm to generate parent vectors and adopt a population size reduction strategy. There are three main differences between the proposed algorithm and the above memetic algorithms: (1) The proposed algorithm performs much more local searches than global searches. (2) The proposed algorithm performs the local search for every individual. (3) The proposed algorithm uses a new and simpler global search method.

In the following sections, the details of the MPCE & SSALS algorithm will be explained. The algorithm is also compared with four state-of-the-art algorithms, namely, SHADE-ILS, MLSHADE-SPA, CBCC-RDG3, and IMLSHADE-SPA.

The main contributions and novelty of this paper can be summarized as follows:

- Proposing a novel memetic algorithm for the LSGO problem
- Using multiparent crossover and SGSO to solve LSGO problem
- Proposing an improved local search algorithm that can be an effective option for LSGO
- Demonstrating that local search-dominated hybrid algorithm can effectively solve the LSGO problems.

The rest of this paper is organized as follows. In Section 2, the most related work to this paper proposed approach is discussed.  Section 3 presents the details of the proposed algorithm.  Section 4 explains the numerical experiments of MPCE & SSALS that are carried out using the CEC′2013 benchmark suite and the performance of MPCE & SSALS compared to four algorithms. Finally, conclusions are made, and further research is discussed in Section 5.

## 2. Related Works

This section is devoted to presenting the related work needed for understanding the MPCE & SSALS algorithm. Memetic algorithms, multiparent crossover, simplified group search optimizer, and MTS are described.

### 2.1. Memetic Algorithms

Moscato [23] first proposed the concept of memetic algorithm in 1989. The memetic algorithm is a combination of population-based global search and individual-based heuristic local search. It suggests an algorithm framework. In this framework, different search strategies are used to construct different memetic algorithms. For example, Genetic algorithms, Differential Evolution, Particle Swarm Optimization, and many others can be used for global search strategy. Hill Climbing, Simulated Annealing, Tabu Search, and others can be used for local search strategy. Memetic algorithms have embraced many forms, employing a wide variety of combinations of population-based heuristics and individual improvement heuristics [25], such as [26–33]. Some of these algorithms based on GA and Tabu Search were studied in [26,27]. The memetic model of PSO and local search was introduced in [28–30]. A Memetic Artificial Bee Colony Algorithm is also reported in [31]. The combination of a backbone-based crossover operator and a multineighborhood simulated annealing procedure was discussed in [32]. In [33], adaptive memetic computing with a GA, DE, and Estimation of Distribution Algorithm synergy was elaborated. It can automatically activate one of the three algorithms to generate offspring.

Memetic algorithms combine the exploration capability of population-based global search with the rapid exploitation capability of local search. The hybridization between global and local search algorithms has been experimentally proven to provide better search performance [33]. Many examples have proved the effectiveness of this strategy, including many difficult problems, such as multimodal optimization [33,34], large-scale global optimization [5–19], combinatorial optimization [32,35], single-objective optimization [36,37], and multiobjective optimization [38,39]. For large-scale global optimization problems, most of the best-performing algorithms were hybrid algorithms combining global and local search (e.g., SHADE-ILS, MLSHADE-SPA, and MOS).

SHADE with an iterative Local Search (SHADE-ILS) is a hybrid algorithm that combines a modern DE algorithm, Success-History-based Adaptive DE (SHADE [40]), with two local search methods. In each iteration, the SHADE is applied to evolve the population of candidate solutions. One of the two local search methods is chosen to improve the current best solution found by SHADE. The local search method's selection is according to the improvement obtained by each of them in the previous phase. A restart mechanism has been incorporated into the algorithm to explore new search space regions when the search gets stagnated.

MLSHADE-SPA is a memetic framework that includes three DE algorithms for global exploration and a modified version of MTS (MMTS) for local exploitation. The three DE algorithms are success history-based differential evolution with linear population size reduction and semiparameter adaptation (LSHADE-SPA), enhanced adaptive differential evolution (EADE) [41], and differential evolution with novel mutation and adaptive crossover strategies (ANDE) [42]. The framework also uses the divide-and-conquer method, which randomly divides the dimensions into groups and solves each group separately.

An improved MLSHADE-SPA (IMLSHADE-SPA) framework was proposed in [11], which replaced the local search method (MMTS) with a new local search method and achieved higher performance.

Multiple Offspring Sampling (MOS) [43] is a framework used to combine different metaheuristic algorithms. The participation ratio for each algorithm is adjusted dynamically according to a given strategy. Due to the different algorithms and strategies to be selected, different MOS versions were proposed in [9,44,45]. Our paper focuses on the MOS [9], the winner in the CEC′2013 competition. In MOS [9], three algorithms are combined: GA, Solis and Wets algorithm [46], and MTS-LS1-Reduced algorithm. These algorithms are executed in sequence, one after the other. The number of candidate solutions to be generated by each algorithm is adjusted dynamically according to the average fitness increment of the newly created individuals [9].

### 2.2. Multiparent Crossover

Evolutionary algorithms (EAs) have been successfully applied to solve many optimization problems. EAs simulate the evolution process of nature. There are three basic operators in EAs: crossover (or recombination), mutation, and selection. The classic crossover operator recombines two parents and generates new offspring. The recombination mechanism determines what parts of each parent are inherited by the child and how this is done. Various crossover operators were proposed for different problems that fit one of the multiple representations for a chromosome [47]. These crossover operators can be categorized into two categories: exchange-based or calculation-based. The first type of operator is generally proposed for binary coding, but it is also suitable for real coding. Some of the crossover operators' examples are One-point Crossover, Two-point Crossover, Uniform Crossover, and so on. For instance, Uniform Crossover randomly determines whether the child's *i*th gene is selected from father 1 or father 2. With these crossover mechanisms, each gene in the offspring is copied from one of the parents. The new offspring's chromosome characteristics are directly inherited from their parents without any changes.

The second category of the crossover operators is generally used for real coding, such as Average Crossover, Parent Centric Crossover, Heuristic Crossover, Simulated Binary Crossover, and so on. In these operators, the value of each offspring's gene is calculated numerically by the parents' genes. For example, Average Crossover generates the *i*th gene of the child by averaging alleles from both parents.

The first category is more in line with the original concept of gene recombination. In some algorithms, such as the DE algorithm, the second category crossover operator is used as a mutation rather than a crossover operator. It can produce new genes that are different from their parents. This paper tends to define the second type of operators as a hybrid of crossover and mutation operations.

Multiparent crossover extends the two-parent crossover operators to recombine more than two parents for generating new offspring. Many multiparent crossovers have been successfully applied to solve various optimization problems and found to be better than traditional crossovers, such as scanning crossover and diagonal crossover [48,49], multiparent simplex crossover [50], multiparent sequential constructive crossover [47], and a novel multiparent order crossover [51].

### 2.3. Simplified Group Search Optimizer

Group Search Optimizer (GSO) is a swarm intelligence algorithm with superior performance for multimodal problems [52].

GSO is inspired by animal searching behaviors and group living theory [52]. It includes three types of members: producer, scrounger, and ranger. During each iteration, the individual with the best fitness value in the group, as a producer, will stop and scan the environment to find resources. The scrounger takes a random walk towards the producer to join the resources. A small number of rangers make a random move to avoid entrapment in local minima.

The Simplified Group Search Optimizer (SGSO) [24] is an improved GSO version. It is more efficient and simpler than the original version. It also shows excellent search performance for large-scale optimization problems. In SGSO, the producer abandons environmental scanning. The scrounger adopts an improved join strategy, which moves towards the best member and other excellent members. The rangers use a simple search method and the ranger's percentage decreases. The SGSO is described as follows:

(1) In a *D*-dimensional search space, the *i*th member at the *k*th iteration has a current position, **x**_*i*,*k*_ ∈ *R*^*D*^.
(2) Group members are sorted by fitness value in ascending order. The best member **x**_best,*k*_, as the producer, does not move in this iteration.
(3) Randomly select 87% of the group members except the producer to perform scrounging. The scroungers move to a new position according to
  (2) $$\begin{array}{c} x_{i,k+1}=x_{i,k}+r_{1}\left(x_{\text{best},k}-x_{i,k}\right)+r_{2}\left(x_{m-\text{best},k}-x_{i,k}\right), \end{array}$$
where ***r***_1_ and ***r***_2_ are uniform random *D*-dimensional vectors in the range (0, 1) and **x**_*m*−best,*k*_ is a member randomly chosen from the top 4 in the group (except **x**_best,*k*_).
(4) The remaining members are rangers, who take a random step according to
  (3) $$\begin{array}{c} x_{i,k+1}=x_{i,k}+r_{3}\cdot f*\text{step}, \end{array}$$
where ***r***_3_ is a standard normal distribution *D*-dimensional vector, step is a constant, representing the basic step size, and ***f*** is a *D*-dimensional Boolean random vector indicating which dimensions will change. The probability of change is set to be 1.2/*D* as given in [24].
(5) ***f*** is calculated by
  (4) $$\begin{array}{c} f_{j}=\left\{\begin{array}{cc} 1, & \text{if rand}\left(1\right)\leq \frac{1.2}{D}\text{ or }j=j_{\text{rand}},\\ 0, & \text{otherwise}, \end{array}\right. \end{array}$$
where *j* ∈ {1,2,…, *D*}, rand(1) is a function that produces a uniform random number in the range (0, 1), and *j*_rand_ is a randomly chosen index ∈ {1,2,…, *D*}, which ensures that at least one component in ***f*** is set to 1.

### 2.4. Multiple Trajectory Search

Multiple trajectory search (MTS) was presented for the large-scale global optimization problem in [10]. It provides three local search methods, where MTS-LS1 is the first and most important one.

MTS-LS1 does search from the first to the last dimension successively. Each dimension is subtracted from the search range (SR) value to see whether the objective function value is improved or not. If it is improved, MTS-LS1 proceeds to search in the next dimension. If it is not improved, the solution is restored, and this dimension is added by 0.5*∗* SR, aiming to see, again, if its value is improved or not. If it is not improved, the solution is restored. Afterward, MTS-LS1 continues to search in the next dimension. SR is initialized to 0.5*∗* (Upper_Bound − Lower_Bound). If all dimensions are not improved, SR will be cut to half. When SR reaches 1*E* − 15, its value will be reset to 0.4*∗* (Upper_Bound − Lower_Bound). MTS-LS1 and its improved versions are used in many algorithms [5,9,12], including the algorithm proposed in this paper.

## 3. Proposed Algorithm

In this section, multiparent Crossover Evolution and Step-Size Adaptive Local Search algorithm will be described. Besides, the proposed hybrid algorithm that combines both of them will be introduced.

### 3.1. Multiparent Crossover Evolution (MPCE)

In MPCE, the population is composed of *D*-dimensional vectors. The number of vectors is called population size, denoted as NP. The initial population is generated with uniformly distributed random numbers. Each member of the population can produce the next generation through mutation and multiparent crossover operation. The *i*th member of the *G*th generation is denoted as ***x***_*i,G*_.

The main characteristics of MPCE are as follows:

(1) The mutation formula is modified from (2) of the SGSO algorithm. The mutant vector is generated according to
  (5) $$\begin{array}{c} v_{i,G}=x_{i,G}+r_{1}\left(x_{\text{best},G}-x_{i,G}\right)+r_{2}\left(x_{p-\text{best},G}-x_{i,G}\right), \end{array}$$
where ***x***_best, *G*_ is the best vector in the *G*th generation, *p*-best is the index of a vector which is randomly chosen from the ranked top 10% vectors in the *G*th generation (except ***x***_best, *G*_), and ***r***_1_ and ***r***_2_ are uniform random vectors in the range (0, 1).
(2) MPCE uses a four-parent crossover operation to produce the next generation. The four parents are ***x***_*i*_, *v*_*i*_ and two excellent individuals randomly selected from the population. The crossover operation could be computed using
  (6) $$\begin{array}{c} x_{ji,G+1}=\left\{\begin{array}{cc} v_{ji,G}, & \text{if }r_{\text{rand}\left(ji\right)}\leq CP1,\\ x_{ja\left(i\right),G}, & \text{if }CP1<r_{\text{rand}\left(ji\right)}\leq CP1+CP2,\\ x_{jb\left(i\right),G}, & \text{if }CP1+CP2<r_{\text{rand}\left(ji\right)}\leq CP1+CP2+CP3,\\ x_{ji,G}, & \text{otherwise,} \end{array}\;\right. \end{array}$$
where *j*∈{1,2,…, *D*}, *a*(*i*) and *b*(*i*)∈{1,2,…,*NP*} are the index of vectors randomly chosen from ranked top 50% vectors in the *G*th generation, CP1, CP2, CP3 ∈ (0,1) are the crossover probability constant of *v*_*i*_, ***x***_a(*i*)_, ***x***_b(*i*)_, respectively, ***r***_rand(*ji*)_ is a uniform random number in the range (0, 1).
The parameters CP1, CP2, and CP3 are determined through experiments and set to 0.3, 0.29, and 0.29, respectively.
(3) The population size decreases during the optimization process. With the ongoing iteration, the vectors in the population tend to be gradually assimilated, where the larger NP is less helpful to improve the search performance. Many algorithms apply the population size linear decrease strategies, such as LSHADE algorithm [53]. Besides, for the MPCE & SSALS algorithm, reducing the population size is conducive to deeper local search. In the beginning, the global search and the local search are performed alternately. NP is reduced by 1, and the worst individual in the population is dismissed every several iterations. When NP is reduced to 4, MPCE global search ends and then only the local search is executed to improve the current best solution.

### 3.2. Step-Size Adaptive Local Search (SSALS)

The basic idea of SSALS derives from MTS-LS1 that is the first local search strategy in the Multiple Trajectory Search (MTS) algorithm. These algorithms are designed for single individuals and can also be used for multiple individuals when combined with other algorithms.

Each dimension of the SSALS algorithm has its basic step size, stored in the vector ***s***. In each iteration, SSALS randomly selects one or more dimensions, multiplies the step size of each dimension by a random number, and adds the product to each dimension. If the new solution is better than the original one, these selected dimensions' step size is multiplied by 2. Otherwise, the solution is restored, and each step size is multiplied by −0.5. The step size is initialized using 0.5*∗* (Upper_Bound − Lower_Bound). The variable *minbs* represents the minimum step size, an adaptive value that is recalculated in each iteration. If the step size's absolute value reaches *minbs*, it will be restored using the initial value.

In the case of multiple individuals, the SSALS algorithm key steps are described as follows.

(1) Choose dimensions to be searched according to
  (7) $$\begin{array}{c} f_{ji,G}=\left\{\begin{array}{cc} 1, & \text{if rand}\left(1\right)<\frac{0.5}{D}+{\left(\frac{0.1*D}{\text{iteration}}\right)}^{2}\text{ or }j=j_{\text{rand}\left(i\right)},\\ 0, & \text{otherwise,} \end{array}\right. \end{array}$$
where *f*_*ji*_ ∈ {0,1} indicates whether the *j*th dimension of the *i*th vector is to be changed, rand(1) is a function that produces a uniform random number in the range (0, 1), *iteration* is the number of iterations, and *j*_rand(*i*)_ ∈ {1,2,…, D} is a randomly chosen index to ensure that ***x***_*i*_ has at least one dimension to participate in the search.
According to (7), the number of dimensions to be searched will rapidly decrease in the iterative process and finally keep at 1.5 per vector on average. This value makes the algorithm has a bit of global search ability in the early stage of the optimization process.
(2) Generate the new solution according to
  (8) $$\begin{array}{c} x_{i,G+1}=x_{i,G}+s_{i,G}\cdot \text{rand}\left(\text{D},1\right)\cdot f_{i,G}, \end{array}$$
where ***s***_*i,G*_ is a vector, representing the basic step size of the *i*th individual in the *G*th generation.
(3) Calculate the variate *minbs.* SSALS defines a *D*×5 matrix ***H***, which is used to store each dimension's last five effective step sizes. The effective step size is defined as
  (9) $$\begin{array}{c} e_{ji,G+1}=\left\{\begin{array}{cc} \left|x_{ji,G+1}-x_{ji,G}\right|, & \text{if }x_{i,G+1}\text{ is better than }x_{i,G}\text{ and }x_{ji,G+1}\neq x_{ji,G},\\ \text{null,} & \text{otherwise,} \end{array}\right. \end{array}$$
If more than one vector is improved in an iteration, and some of these vectors' same dimension is changed, save the average effective step size of this dimension into ***H***.
The formula for calculating *minbs* is given in
  (10) $$\begin{array}{c} {\text{minb}}_{s}G=\text{min}\left(0.1,\min\left(\text{mean}\left(H,2\right)\right)\right). \end{array}$$
(4) Update the basic step size according to
  (11) $$\begin{array}{c} s_{ji,G+1}=\left\{\begin{array}{cc} s_{ji,G}\times \left(-0.5\right), & \text{if }x_{i,G}\text{ is better than }x_{i,G+1},\text{ and }f_{ji,G}=1,\\ s_{ji,G}\times 2, & \text{if }x_{i,G}\text{ is not better than }x_{i,G+1},\text{ and }f_{ji,G}=1,\\ s_{ji,G}, & \text{otherwise.} \end{array}\right. \end{array}$$

### 3.3. Hybrid Algorithm: MPCE and SSALS

MPCE & SSALS is a memetic algorithm based on MPCE and SSALS, presented in Algorithm 1. The hybrid strategy is to perform one global search iteration after a certain number of local search iterations. The constant *I*_GS_ indicates the interval of global search. Also, the constant *I*_NPD_ refers to the decreased interval of NP. In other words, NP is subtracted by 1 for each *I*_NPD_ iteration. When NP is reduced to 4, the global search ends, and only the local search is performed to improve the current best solution. The parameters *I*_GS_ and *I*_NPD_ are determined by experiments in which they are set to 40 and 100, respectively.

MPCE & SSALS performs a boundary check on each new individual generated, and all values outside the boundary will be reset to random numbers within this boundary. The pseudocodes of the proposed algorithms are given in Algorithm 1.

## 4. Experimentation

A set of 15 benchmark functions proposed in the CEC 2013 special session on large-scale global optimization was used to study the MPCE & SSALS performance. These functions are divided into four categories according to the degree of separability. f1–f3 belong to fully separable functions, f4–f11 are partially separable functions, f12–f14 belong to overlapping functions, and f15 is classified as fully nonseparable functions. A detailed description of each of these benchmark functions is given in [20].

MPCE & SSALS performed 25 times for each benchmark function. All tests were completed using MATLAB R2019a. The dimension *D* of all functions is 1000, except that f13 and f14 are 905. The stopping criterion was a fixed number of fitness evaluations (FEs). The Max_NFE was set to be 3.0*E* + 6, and the program terminates when Max_NFE is reached. The initial value of NP was set to 100, CP1 = 0.3, CP2 = 0.29, CP3 = 0.29, *I*_NPD_ = 100, and *I*_GS_ = 40. The statistical results including the best, the worst, the median, the mean, and the standard deviation computed over 25 runs are shown in Table 1.

### 4.1. Influence of the Different Components

In this section, experiments were conducted to observe the influence of the different components. For each test, Table 2 lists the average results of 25 independent runs. Wilcoxon signed-rank test with the significance level of 5% was used for statistical analysis. The “>,” “<,” and “=” mean “significantly better,” “significantly worse,” and “no significant difference,” respectively. The last row of Table 2 shows the times of win/tie/loss (w/*t*/l) in the pairwise comparison.

To observe the individual effect of both Multiparent Crossover Evolution and Step-Size Adaptive Local Search, experiments were executed on the two algorithms, respectively. As shown in Table 2, the optimization performance of SSALS is significantly better than that of MPCE on most of the functions, indicating that local searches contribute more to the hybrid algorithm.

The influence of the number of parents was also studied. In the proposed algorithm, CP2 and CP3 are the crossover probability constants of parent 2 and parent 3, respectively. CP2 = 0 indicates that parent 2 does not participate in the evolutionary operation, so is CP3. In one test, CP2 was set to 0, indicating that the three-parent crossover operation was used. In another test, CP2 and CP3 were both set to 0, which means that a two-parent crossover operation was applied. The other settings are considered the same as in Table 1. According to the results, increasing the number of parents affects f5, f6, f9, and f10, but it has no significant difference on other functions. In general, it is beneficial and harmless.

In addition, to verify the improvement effect of SSASL, the same experiments were performed in identical conditions with replacing MTS-LS1 with SSALS. In the comparison test between SSALS with MTS-LS1, it is clear that SSALS is significantly better than MTS-LS1 on all 15 functions, demonstrating that the optimization performance of SSALS is significantly higher than that of MTS-LS1.

### 4.2. Parameter Analysis

Major parameters of the MPCE & SSALS are *I*_NPD_ and I_GS_. For each *I*_NPD_ iteration, population size (NP) is subtracted from 1. When NP is reduced to 4, the population-based search ends, which means only the individual-based search is performed to improve the best solution. Therefore, a smaller *I*_NPD_ means fewer population searches and more single individual searches. *I*_GS_ indicates the number of iterations between two global searches, and a smaller I_GS_ represents more global searches and fewer local searches. Different *I*_NPD_ and *I*_GS_ are studied in this section. MPCE & SSALS performed 25 times for each combination. Wilcoxon signed-rank test was used for statistical analysis.

To find the appropriate *I*_NPD_ and *I*_GS_ value, three CEC′2013 benchmark functions f3, f7, and f15 are studied in the tests with *I*_NPD_ value varying from 50 to 500 and *I*_GS_ value varying from 20 to 200, respectively. The other parameters use the same settings as in Table 1. Algorithm performances by adopting different *I*_NPD_ and *I*_GS_ values on f3, f7, and f15 are shown in Figures 1(a), 1(b), and 1(c), and Figures 2(a), 2(b), and 2(c), respectively. The horizontal axis represents the respective parameter settings while the vertical axis shows the obtained logarithm value of mean FEs. As shown in Figures 1 and 2, the best result was obtained when *I*_NPD_ = 100 and *I*_GS_ = 40.

The test results of some different combinations of *I*_NPD_ and *I*_GS_ with {50,40}, {100,40}, {200,40}, {100,20}, and {100,80} in 15 benchmark functions are shown in Table 3. Results shown in bold indicate the final selected parameters. When fixing *I*_GS_ value at 40, *I*_NPD_ = 100 significantly outperforms *I*_NPD_ = 50 in 5 functions and is outperformed by *I*_NPD_ = 50 in 1 function, while other the 9 functions have no significant difference. *I*_NPD_ = 100 significantly outperforms *I*_NPD_ = 200 in 7 functions and is outperformed by *I*_NPD_ = 50 in 2 functions, which indicate that the best overall optimization performance is *I*_NPD_ = 100. When *I*_NPD_ is fixed at 100, *I*_GS_ = 40 significantly outperforms *I*_GS_ = 20 and *I*_GS_ = 80 in 2 and 3 functions, respectively. There is no significant difference in other functions, which means that the best optimization performance is *I*_GS_ = 40. As shown in Table 3, MPCE-SSALS with *I*_NPD_ = 100 and *I*_GS_ = 40 significantly outperforms the other parameter settings. It is also observed that the best parameter values of different test functions may be different; for example, the best parameter for f3 and f6 is *I*_NPD_ = 200 and *I*_GS_ = 40. This suggests that it is a good choice to set the parameter values to 100 and 40 in general, but for a specific problem, better parameter values can be determined by experiments.

In addition, when *I*_NPD_ = 100 and *I*_GS_ = 40, the FEs of global search and local search are 12524 and 2987476, respectively, which indicates that the proposed algorithm is mainly based on local search.

### 4.3. Comparison with the Reference Algorithm

MPCE & SSALS was compared with other state-of-the-art algorithms, including SHADE-ILS [12], MLSHADE-SPA [5], CBCC-RDG3 [17], and IMLSHADE-SPA [11]. Among them, SHADE-ILS, CBCC-RDG3, and MLSHADE-SPA were currently the top three algorithms in the CEC LSGO competitions, and IMLSHADE-SPA is an improved version of MLSHADE-SPA.

To compare these algorithms' performances on the CEC′2013 function suite, the average ranking of each algorithm was calculated. For a fair comparison, the other four algorithms' experimental data and supplementary material are directly taken from their original papers. Wilcoxon signed-rank test (significance level = 0.05) is utilized for pairwise comparison of these five algorithms. The place of each algorithm on each function is calculated according to the Wilcoxon rank tests. The comparison results and ranking are listed in Table 4. The best results for each benchmark function are distinguished by bold font.

As shown in Table 4, MPCE & SSALS is the one with the best performance among these algorithms. SHADE-ILS and IMLSHADE-SPA rank second and third, respectively. Compared with SHADE-ILS, MLSHADE-SPA, CBCC-RDG3, and IMLSHADE-SPA, MPCE & SSALS won in 8, 9, 10, and 7 functions but lost in 5, 4, 5, and 3 functions, respectively. For the 15 benchmark functions, MPCE & SSALS obtained 8 best results, while SHADE-ILS, MLSHADE-SPA, CBCC-RDG3, and IMLSHADE-SPA obtained 3, 4, 5, and 3 best results, respectively. For fully separable functions, MPCE & SSALS performs the best. CBCC-RDG3 achieves the best on partially separable functions. For overlapping functions and fully nonseparable functions, MPCE & SSALS and SHADE-ILS give the best results.

Figure 3 shows the convergence curve of MPCE & SSALS, SHADE-ILS, MLSHADE-SPA, CBCC-RDG3, and IMLSHADE-SPA in 15 benchmark functions.

As shown in the figure, the results could be summarized as follows:

- MPCE & SSALS has a faster convergence rate than IMLSHADE-SPA in the functions f1–f3, f5–f7, f9, and f13–f15, but it has a slower convergence rate than IMLSHADE-SPA in the functions f4, f8, and f10–f12.
- MPCE & SSALS has a faster convergence rate than SHADE-ILS in the functions f2, f3, f5, f6, f9, f10, and f15, but it has a slower convergence rate than SHADE-ILS in the functions f1, f4, f7, f8, and f11–f14.
- MPCE & SSALS has a faster convergence rate than MLSHADE-SPA in f1, f5, f6, f7, f9, and f13–f15 functions; however, it has a slower convergence rate than MLSHADE-SPA in f3, f4, f8, f10, and f12 functions.
- MPCE & SSALS has a faster convergence rate than CBCC-RDG3 in f2, f3, f6, f10, and f15 functions, but it has a slower convergence rate than CBCC-RDG3 in f4, f7, f8, f11, and f13 functions.

The convergence rate of MPCE & SSALS, in general, is faster than that that of MLSHADE-SPA and IMLSHADE-SPA, but it has a similar convergence rate to CBCC-RDG3 and SHADE-ILS. However, MPCE & SSALS is the simplest one among these algorithms.

### 4.4. Results Discussion

The excellent results of MPCE & SSALS mainly benefit from the following factors:

1. The multiparent strategy used in this paper enables each offspring to inherit genes from multiple excellent individuals. It not only increases the offspring diversity, but also moves the algorithm quicker towards better solutions.
2. SSALS effectively improves MTS-LS1, which enhanced the local search performance significantly. Each dimension has its own basic step size that can be adjusted to accommodate the different effects of each dimension on the function. In addition, the minimum step size affects the search accuracy. If a large number of high-precision searches (very small step size) are carried out in the early stage of the algorithm, it will waste an amount of calculation and easily fall into the local minima. According to the current search results, gradual improvement to the search accuracy can avoid excessive search in the early stage of the algorithm. Similarly, in the late stage of the algorithm, the most promising position can be searched with high precision.
3. More local searches are performed in the algorithm. The proposed algorithm performs much more local searches than global searches. This enhances the exploitation capability of the algorithm in the search space.
4. Population decrease strategy is used in MPCE & SSALS. At the beginning of the algorithm, a large population size is conducive to improving the exploration ability. With the optimization process, individual differences are minimized, and the advantages of a large population are also reduced. Gradually reducing the population size is helpful to enhance the exploitation ability.
5. The memetic algorithm framework is used to combine the multiparent strategy, SGSO and SSALS, to work together. The memetic algorithm framework balances the exploration ability of global search and the exploitation ability of local search; thus, it has been widely used in LSGO problems. The SGSO algorithm also performs well in LSGO problems.

## 5. Conclusions

In this paper, a memetic algorithm MPCE & SSALS based on multiparent crossover evolution and step-size adaptive local search is proposed for LSGO problem. The MPCE strategy is used for global exploration, and the SSALS method is applied for local exploitation. In the early stage of algorithm execution, the global search and the local search are performed interchangeably, and the population size is gradually reduced to 1. In the later stage, only the local search is executed to improve the final solution. Local search is performed during the whole process, and the execution times of local search is far more than that of global search. A set of 15 benchmark functions was used to evaluate the performance of the MPCE & SSALS algorithm. According to the experimental data, the overall performance of the MPCE & SSALS algorithm performs better than the other four state-of-the-art algorithms. The experimental results also indicate that the performance of SSALS is significantly higher than that of MTS-LS1, and the local search-dominated hybrid algorithm can effectively solve the LSGO problem.

On the other hand, the experiment analysis reveals that the multiparent crossover strategy can only improve the optimization effect of certain test functions while having no discernible impact on others. Among the four parents in the crossover operation, three individuals are selected from the previous generation of the population. The source of parents is relatively single. The advantages of multiparenting were not fully used. In the future, it is possible to add new parent generation methods, such as using PSO to generate one of the parents. This paper demonstrated that multiparent crossover evolution combined with local search is an effective algorithm framework to address the LSGO problem. A possible extension to this paper is to examine new parent generation techniques or local search strategies that improve the algorithm's performance.

## Figures and Tables

**Figure 1:** Comparison of different *I*_NPD_ values. (a) f3. (b) f7. (c) f15.

**Figure 2:** Comparison of different *I*_GS_ values. (a) f3. (b) f7. (c) f15.

**Figure 3:** Convergence curves on f1–f15. (a) f1. (b) f2. (c) f3. (d) f4. (e) f5. (f) f6. (g) f7. (h) f8. (i) f9. (j) f10. (k) f11. (l) f12. (m) f13. (n) f14 (o) f15.

**Algorithm 1:** Multiparent Crossover Evolution and Step-Size Adaptive Local Search algorithm.

**Table 1:** MPCE & SSALS statistical result on the CEC′2013 LSGO functions, *D* = 1000, FEs = 3.0*E* + 06.

Milestone	Category	f1	f2	f3	f4	f5	f6	f7	f8	f9	f10	f11	f12	f13	f14	f15
1.2*E* + 05	Mean	6.27*E* + 09	1.73*E* + 04	1.94*E* + 01	5.47*E* + 11	1.00*E* + 07	2.95*E* + 05	7.26*E* + 09	1.01*E* + 16	7.38*E* + 08	1.61*E* + 06	1.31*E* + 12	2.30*E* + 11	2.96*E* + 11	2.74*E* + 12	2.62*E* + 08
6.0*E* + 05	Mean	7.90*E* + 01	7.95*E* + 02	1.07*E* + 00	3.99*E* + 10	1.18*E* + 06	7.46*E* + 02	2.32*E* + 08	2.24*E* + 15	9.02*E* + 07	5.00*E* + 04	4.11*E* + 10	2.83*E* + 03	4.65*E* + 09	7.84*E* + 10	7.56*E* + 06
3.0*E* + 06	Best	0.00*E* + 00	1.57*E* − 26	3.34*E* − 13	1.61*E* + 09	9.32*E* + 05	3.34*E* + 01	2.64*E* + 03	6.70*E* + 13	6.89*E* + 07	7.40*E* + 03	2.45*E* + 05	1.48*E* − 02	1.44*E* + 05	4.95*E* + 06	5.09*E* + 05
	Median	3.94*E* − 28	9.95*E* − 01	3.59*E* − 13	3.29*E* + 09	1.22*E* + 06	7.20*E* + 02	4.10*E* + 03	1.86*E* + 14	8.94*E* + 07	2.37*E* + 04	2.63*E* + 06	1.31*E* + 01	1.36*E* + 06	5.41*E* + 06	5.86*E* + 05
	Worst	1.51*E* − 26	3.98*E* + 00	3.77*E* − 13	5.55*E* + 09	1.46*E* + 06	1.40*E* + 03	7.27*E* + 03	3.00*E* + 14	1.15*E* + 08	1.43*E* + 05	1.51*E* + 07	2.24*E* + 02	2.14*E* + 07	6.27*E* + 06	6.49*E* + 05
	Mean	1.53*E* − 27	1.35*E* + 00	3.59*E* − 13	3.56*E* + 09	1.18*E* + 06	7.46*E* + 02	4.39*E* + 03	1.84*E* + 14	9.02*E* + 07	4.98*E* + 04	3.32*E* + 06	5.85*E* + 01	3.56*E* + 06	5.46*E* + 06	5.80*E* + 05
	Std	3.24*E* − 27	1.34*E* + 00	9.94*E* − 15	9.66*E* + 08	1.38*E* + 05	2.81*E* + 02	1.40*E* + 03	4.97*E* + 13	1.21*E* + 07	4.81*E* + 04	3.49*E* + 06	6.71*E* + 01	5.66*E* + 06	3.42*E* + 05	3.59*E* + 04

**Table 2:** Comparison of different components on the CEC′2013 LSGO functions, *D* = 1000, FEs = 3.0*E* + 06 (with Wilcoxon test, *α* = 0.05).

Fun	MPCE		SSALS		MPCE & SSALS		MPCE & SSALS		MPCE & MTS-LS1		MPCE & SSALS
	Four parents				Two parents		Three parents		Four parents		Four parents
f1	3.50*E* + 10	<	1.53*E* − 27	=	1.48*E* − 27	=	2.49*E* − 27	=	3.24*E* − 25	<	1.53*E* − 27
f2	2.63*E* + 04	<	5.97*E* − 01	=	1.52*E* + 00	=	1.39*E* + 00	=	3.28*E* + 02	<	1.35*E* + 00
f3	2.01*E* + 01	<	1.32*E* + 01	<	3.42*E* − 13	=	3.59*E* − 13	=	1.65*E* − 12	<	3.59*E* − 13
f4	1.03*E* + 12	<	3.67*E* + 09	=	3.51*E* + 09	=	3.70*E* + 09	=	1.52*E* + 10	<	3.56*E* + 09
f5	6.75*E* + 06	<	2.24*E* + 07	<	1.45*E* + 06	<	1.31*E* + 06	<	2.00*E* + 06	<	1.18*E* + 06
f6	6.43*E* + 05	<	9.84*E* + 05	<	5.44*E* + 04	<	3.98*E* + 03	<	2.53*E* + 05	<	7.46*E* + 02
f7	1.74*E* + 10	<	1.29*E* + 05	<	6.07*E* + 03	=	5.20*E* + 03	=	1.30*E* + 07	<	4.39*E* + 03
f8	2.86*E* + 16	<	3.14*E* + 14	<	1.60*E* + 14	=	1.32*E* + 14	=	1.46*E* + 15	<	1.84*E* + 14
f9	5.97*E* + 08	<	1.52*E* + 09	<	1.13*E* + 08	<	9.60*E* + 07	=	1.50*E* + 08	<	9.02*E* + 07
f10	1.86*E* + 07	<	8.90*E* + 07	<	1.03*E* + 05	<	6.51*E* + 04	=	8.14*E* + 06	<	4.98*E* + 04
f11	4.42*E* + 12	<	1.15*E* + 07	<	3.76*E* + 06	=	3.65*E* + 06	=	1.41*E* + 10	<	3.32*E* + 06
f12	7.66*E* + 11	<	4.98*E* + 01	>	9.40*E* + 01	=	4.45*E* + 01	=	8.07*E* + 02	<	5.85*E* + 01
f13	1.61*E* + 12	<	4.06*E* + 07	<	2.52*E* + 06	=	2.19*E* + 06	=	1.19*E* + 09	<	3.56*E* + 06
f14	4.99*E* + 12	<	7.65*E* + 06	<	5.35*E* + 06	=	5.51*E* + 06	=	1.65*E* + 10	<	5.46*E* + 06
f15	4.83*E* + 13	<	8.58*E* + 05	<	5.93*E* + 05	=	5.76*E* + 05	=	4.26*E* + 07	<	5.80*E* + 05
*w/t/l*	15/0/0		11/3/1		4/11/0		2/13/0		15/0/0		/

**Table 3:** Optimization results of MPCE-SSALS with different combinations of parameters *I*_NPD_ and *I*_GS_ (with Wilcoxon test, *α* = 0.05).

Fun	*I*_NPD_ = 100, *I*_GS_ = 40	*I*_NPD_ = 50, *I*_GS_ = 40		*I*_NPD_ = 200, *I*_GS_ = 40		*I*_NPD_ = 100, *I*_GS_ = 20		*I*_NPD_ = 100, *I*_GS_ = 80	
f1	1.53*E* − 27	=	5.95*E* − 28	=	1.22*E* − 27	=	5.78*E* − 28	=	2.15*E* − 27
f2	1.35*E* + 00	=	4.98*E* − 01	=	3.48*E* + 00	=	1.09*E* + 00	=	1.31*E* + 00
f3	3.59*E* − 13	>	3.80*E* − 13	=	3.61*E* − 13	=	3.62*E* − 13	=	3.67*E* − 13
f4	3.56*E* + 09	=	3.14*E* + 09	>	5.12*E* + 09	=	3.83*E* + 09	=	3.41*E* + 09
f5	1.18*E* + 06	>	1.43*E* + 06	=	1.20*E* + 06	=	1.17*E* + 06	>	1.51*E* + 06
f6	7.46*E* + 02	>	5.36*E* + 03	<	3.52*E* + 02	=	7.15*E* + 02	>	4.93*E* + 03
f7	4.39*E* + 03	=	3.97*E* + 03	>	1.31*E* + 04	=	5.46*E* + 03	=	5.61*E* + 03
f8	1.84*E* + 14	=	1.58*E* + 14	=	1.91*E* + 14	=	1.74*E* + 14	=	1.58*E* + 14
f9	9.02*E* + 07	>	1.13*E* + 08	=	8.83*E* + 07	=	8.47*E* + 07	>	1.11*E* + 08
f10	4.98*E* + 04	>	1.42*E* + 05	<	2.08*E* + 04	=	4.03*E* + 04	=	8.12*E* + 04
f11	3.32*E* + 06	=	1.25*E* + 06	>	6.65*E* + 06	=	4.61*E* + 06	=	5.06*E* + 06
f12	5.85*E* + 01	<	3.20*E* + 01	>	2.71*E* + 02	>	1.45*E* + 02	=	6.90*E* + 01
f13	3.56*E* + 06	=	2.06*E* + 06	>	1.09*E* + 07	=	2.34*E* + 06	=	4.06*E* + 06
f14	5.46*E* + 06	=	5.30*E* + 06	>	7.70*E* + 06	=	5.45*E* + 06	=	5.47*E* + 06
f15	5.80*E* + 05	=	5.55*E* + 05	>	7.01*E* + 05	>	6.19*E* + 05	=	6.01*E* + 05
*w/t/l*	—	5/9/1		7/6/2		2/13/0		3/12/0	

**Table 4:** Experimental comparisons between MPCE & SSALS and state-of-the-art algorithms on the CEC′2013 LSGO functions, *D* = 1000, FEs = 3.0*E* + 06 (with Wilcoxon test, *α* = 0.05).

Fun	MPCE & SSALS		SHADE-ILS			MLSHADE-SPA			CBCC-RDG3			IMLSHADE-SPA		
	Mean (std)	Place	Mean (std)		Place	Mean (std)		Place	Mean (std)		Place	Mean (std)		Place
f1	**1.53*E* − 27** (3.24*E* − 27)	1	>	2.69*E* − 24 (1.35*E* − 23)	2	>	1.94*E* − 22 (4.79*E* − 22)	3	>	1.14*E* − 18 (1.27*E* − 19)	4	>	4.97*E* − 11 (5.35*E* − 11)	5
f2	**1.35*E* + 00** (1.34*E* + 00)	1	>	1.00*E* + 03 (8.90*E* + 01)	3	>	7.89*E* + 01 (9.69*E* + 00)	2	>	2.31*E* + 03 (1.06*E* + 02)	4	>	4.65*E* + 03 (3.10*E* + 02)	5
f3	3.59*E* − 13 (9.94*E* − 15)	2	>	2.01*E* + 01 (1.12*E* − 02)	4	<	**9.96*E* − 14** (7.91*E* − 15)	1	>	2.04*E* + 01 (5.95*E* − 02)	5	>	2.28*E* + 00 (1.21*E* − 01)	3
f4	3.56*E* + 09 (9.66*E* + 08)	5	<	1.48*E* + 08 (8.72*E* + 07)	2	<	6.90*E* + 08 (4.41*E* + 08)	4	<	**4.29*E* + 04** (7.21*E* + 04)	1	<	3.78*E* + 08 (1.96*E* + 08)	3
f5	**1.18*E* + 06** (1.38*E* + 05)	1	>	1.39*E* + 06 (2.03*E* + 05)	2	>	1.80*E* + 06 (2.34*E* + 05)	3.5	>	2.04*E* + 06 (3.13*E* + 05)	5	>	1.75*E* + 06 (2.07*E* + 05)	3.5
f6	**7.46*E* + 02** (2.81*E* + 02)	1.5	>	1.02*E* + 06 (1.19*E* + 04)	5	=	**1.40*E* + 03** (2.39*E* + 03)	1.5	>	1.00*E* + 06 (2.48*E* + 04)	4	>	3.67*E* + 03 (2.75*E* + 03)	3
f7	4.39*E* + 03 (1.40*E* + 03)	3.5	<	7.41*E* + 01 (5.46*E* + 01)	2	>	5.31*E* + 04 (1.96*E* + 04)	5	<	**1.71*E* − 21** (2.39*E* − 22)	1	=	4.90*E* + 03 (4.25*E* + 03)	3.5
f8	1.84*E* + 14 (4.97*E* + 13)	5	<	3.17*E* + 11 (3.06*E* + 11)	2	<	9.77*E* + 12 (5.53*E* + 12)	3.5	<	**7.11*E* + 03** (2.30*E* + 03)	1	<	5.40*E* + 12 (5.30*E* + 12)	3.5
f9	**9.02*E* + 07** (1.21*E* + 07)	1	>	1.64*E* + 08 (1.57*E* + 07)	3.5	>	1.61*E* + 08 (1.94*E* + 07)	3.5	>	1.57*E* + 08 (2.90*E* + 07)	3.5	>	1.63*E* + 08 (2.01*E* + 07)	3.5
f10	4.98*E* + 04 (4.81*E* + 04)	3	>	9.18*E* + 07 (6.93*E* + 05)	4.5	<	**6.56*E* + 02** (2.40*E* + 02)	1.5	>	9.16*E* + 07 (2.18*E* + 06)	4.5	<	**4.95*E* + 02** (1.04*E* + 02)	1.5
f11	3.32*E* + 06 (3.49*E* + 06)	3.5	<	5.11*E* + 05 (2.25*E* + 05)	2	>	4.04*E* + 07 (1.98*E* + 07)	5	<	**2.18*E* − 13** (1.02*E* − 12)	1	=	2.00*E* + 06 (1.94*E* + 06)	3.5
f12	**5.85*E* + 01** (6.71*E* + 01)	2.5	=	**6.18*E* + 01** (1.04*E* + 02)	2.5	=	**1.04*E* + 02** (7.64*E* + 01)	2.5	>	7.00*E* + 02 (1.46*E* + 02)	5	=	**1.08*E* + 02** (8.62*E* + 01)	2.5
f13	3.56*E* + 06 (5.66*E* + 06)	3.5	<	**1.00*E* + 05** (7.19*E* + 04)	1.5	>	7.21*E* + 07 (4.99*E* + 07)	5	<	**6.43*E* + 04** (4.40*E* + 04)	1.5	=	3.05*E* + 06 (2.11*E* + 06)	3.5
f14	**5.46*E* + 06** (3.42*E* + 05)	1.5	>	5.76*E* + 06 (3.76*E* + 05)	3	>	1.52*E* + 07 (3.08*E* + 06)	4	>	1.65*E* + 09 (1.33*E* + 09)	5	=	**5.44*E* + 06** (5.44*E* + 05)	1.5
f15	**5.80*E* + 05** (3.59*E* + 04)	1.5	=	**6.25*E* + 05** (2.40*E* + 05)	1.5	>	2.76*E* + 07 (9.01*E* + 06)	5	>	2.30*E* + 06 (2.17*E* + 05)	4	>	1.23*E* + 06 (5.98*E* + 05)	3
*w/t/l*	/		8/2/5			9/2/4			10/0/5			7/5/3		
Avg. R of f1–f3	1.33		3.00			2.00			4.33			4.33		
Avg. R of f4–f11	2.94		2.88			3.44			2.63			3.13		
Avg. R of f12–f15	2.25		2.13			4.13			3.88			2.63		
Avg. R	2.43		2.70			3.33			3.30			3.23		
Ranking	1		2			5			4			3		

## Data Availability

The source code and experimental data of MPCE & SSALS can be requested from yydzhwf@xnu.edu.cn.
